RETRACTED

# The Carboxy-terminus of BAK1 regulates kinase activity and is required for normal growth of *Arabidopsis*

**DOI:** 10.3389/fpls.2014.00016

**Published:** 2014-02-04

**Authors:** Man-Ho Oh, Xuejun Wang, Sang Yeol Kim, Xia Wu, Steven D. Clouse, Steven C. Huber

**Affiliations:** ^1^Department of Plant Biology, University of IllinoisUrbana, IL, USA; ^2^Department of Biological Science, College of Biological Sciences and Biotechnology, Chungnam National UniversityDaejeon, South Korea; ^3^Department of Genome Sciences, University of WashingtonSeattle, WA, USA; ^4^Department of Horticultural Science, NC State UniversityRaleigh, NC, USA; ^5^United States Department of Agriculture, Agricultural Research ServiceUrbana, IL, USA

**Keywords:** brassinosteroid, BAK1, BRI1, domain, phosphotyrosine, protein–peptide interaction

## Abstract

Binding of brassinolide to the brassinosteroid-insenstive 1(BRI1) receptor kinase promotes interaction with its co-receptor, BRI1-associated receptor kinase 1 (BAK1). Juxtaposition of the kinase domains that occurs then allows reciprocal transphosphorylation and activation of both kinases, but details of that process are not entirely clear. In the present study we show that the carboxy (C)-terminal polypeptide of BAK1 may play a role. First, we demonstrate that the C-terminal domain is a strong inhibitor of the transphosphorylation activity of the recombinant BAK1 cytoplasmic domain protein. However, recombinant BAK1 lacking the C-terminal domain is unable to transactivate the peptide kinase activity of BRI1 *in vitro*. Thus, the C-terminal domain may play both a positive and negative role. Interestingly, a synthetic peptide corresponding to the full C-terminal domain (residues 576–615 of BAK1) interacted with recombinant BRI1 *in vitro*, and that interaction was enhanced by phosphorylation at the Tyr-610 site. Expression of a BAK1 C-terminal domain truncation (designated BAK1-ΔCT-Flag) in transgenic *Arabidopsis* plants lacking endogenous *bak1* and its functional paralog, *bkk1*, produced plants that were wild type in appearance but much smaller than plants expressing full-length BAK1-Flag. The reduction in growth may be attributed to a partial inhibition of BR signaling *in vivo* as reflected in root growth assays but other factors are likely involved as well. Our working model is that *in vivo*, the inhibitory action of the C-terminal domain of BAK1 is relieved by binding to BRI1. However, that interaction is not essential for BR signaling, but other aspects of cellular signaling are impacted when the C-terminal domain is truncated and result in inhibition of growth. These results increase the molecular understanding of the C-terminal domain of BAK1 as a regulator of kinase activity that may serve as a model for other receptor kinases.

RETRACTED

## INTRODUCTION

Plants contain a large family of receptor-like kinases that are structurally similar to animal receptor kinases and consist of an extracellular domain connected by a single-pass transmembrane domain to the cytoplasmic domain of the protein. The cytoplasmic polypeptide contains a protein kinase domain that is flanked by an N-terminal juxtamembrane domain and C-terminal polypeptide (Shiu and Bleecker, 2001). Animal receptor kinases are usually tyrosine kinases whereas the plant receptor kinases are classified as Ser/Thr kinases on the basis of sequence analysis, but recent work suggests that at least some are dual-specificity kinases that can also autophosphorylate on tyrosine residues (Karlova et al., 2009; Oh et al., 2009a,b, 2011, 2012). The model for plant receptor kinase signaling is based on studies with the receptor kinase, BRI1, and its co-receptor, BAK1, that together function in brassinosteroid (BR) signaling. Current thinking is that binding of the steroid ligand to the extracellular domain of BRI1 (Kinoshita et al., 2005) allows docking of the co-receptor, BAK1, initially through interactions of their leucine-rich repeat extracellular domains (Hothorn et al., 2011; She et al., 2011). Recent studies with recombinant extracellular domains of BRI1 and SERK1 structurally characterized a BRI1-BL-SERK1 complex that forms an integral part of the BRI1 ligand-binding pocket (Santiago et al., 2013). However, in the context of the full-length proteins, it is likely that interactions between other domains also contribute to signaling. For example, the recombinant cytoplasmic domains of BRI1 and BAK1 interact *in vitro* (Li et al., 2002) suggesting that several regions of the receptor and co-receptor may contribute to the specificity and strength of the overall interaction. However, whether simple proximity can explain the reciprocal kinase activation that occurs (Wang et al., 2008) is not known.

Although the kinase domain contains the structures and residues required for phosphoryl transfer from ATP to peptide or protein substrates, the flanking domains often play an important regulatory role and that function can be modulated by phosphorylation of residues within the domains. For example with BRI1, the juxtamembrane domain is an activator of the kinase domain (Oh et al., 2009b, 2012); when the juxtamembrane domain is truncated, autophosphorylation of recombinant BRI1 protein is completely inhibited. In the full-length BRI1 cytoplasmic domain protein, the activating role of the juxtamembrane domain of BRI1 is attenuated by phosphorylation of Tyr-831 (Oh et al., 2009b). In contrast, the BRI1 C-terminal polypeptide is an inhibitor of kinase activity (Wang et al., 2005b; Oh et al., 2009b), and its removal from BRI1 expressed in transgenic plants leads to a hyperactive receptor (Wang et al., 2005b). In the full-length BRI1 protein *in vivo*, it is thought that the inhibitory role of the C-terminal polypeptide can be relieved by phosphorylation of several sites located within the sequence (Wang et al., 2005b). However, little is known about the role of flanking domains with other receptor kinases, and in particular, whether and how the flanking domains may contribute to receptor kinase activity and the overall receptor:co-receptor interaction.

RETRACTED

In the present study, we show that the C-terminal domain of BAK1 inhibits the transphosphorylation activity of BAK1 but is essential for BAK1 to activate BRI1 activity *in vitro*. However, the C-terminal domain is not essential for BR signaling *in vivo* suggesting that other mechanisms provide proper positioning so that the kinase domains of BRI1 and BAK1 can effectively transphosphorylate and activate the signaling cascade. It is also interesting that in the absence of the C-terminal domain of BAK1 plant growth is significantly inhibited suggesting that other (presently unknown) factors are affected by removal of the C-terminal domain. Overall, the results establish an important role for the C-terminal domain of BAK1 and perhaps other receptor kinases as well.

## MATERIALS AND METHODS

### PLANT GROWTH AND TRANSFORMATION

*Arabidopsis thaliana* ecotype Ws-2 was the background for the *bri1-5* mutant and Col-0 was the background for transgenics in the null *bak1-4 bkk1* mutant background. Expression of BAK1::BAK1-Flag (wild type and site-directed mutants) in the *bak1-4 bkk1-1* double mutant background was achieved by transforming the viable heterozygous *BAK1-4 /bkk1-1 bkk1-1* (He et al., 2007) with the pBIB-Hyg-PK1-BAK1-Flag construct and screening for homozygous *bak1-4 bkk1-1* double mutants expressing the transgene as described (Wang et al., 2008). PK1 refers to the native promoter of BAK1 located in the 1.7 Kb sequence upstream of the gene. All site-directed mutants were produced using the Quik Change XL Site-Directed Mutagenesis Kit (Stratagene, La Jolla, CA, USA) and a full-length BAK1 cDNA with C-terminal Flag epitope tag as template. As specified, serial truncations of the C-terminal domain were made by sequentially removing five amino acid segments between residues 615 and 580. In addition, the cDNA lacking the complete C-terminal domain was used to produce directed mutants with the following substitutions: Y304F, Y363F, Y365F, Y403F, Y443F, Y463F, and Y478F. All constructs were sequenced in both directions to verify specific mutations and lack of additional mutations.

RETRACTED

Seeds were surface sterilized, kept at 4°C for 2 days, and then sown on germination medium [1/2 strength Murashige and Skoog salt and vitamins medium (PhytoTechnology Laboratories, Lenexa, KS, USA), supplemented with 0.8% (w/v) agar, 30 mg L^-^^1^ hygromycin B (Sigma-Aldrich, St. Louis, MO, USA) and 2% (w/v) sucrose, pH 5.7]. For phenotypic analysis between plants expressing BAK1-Flag and BAK1-ΔCT-Flag, plates containing half-strength MS medium (0.8% agar) were kept at 22°C with an 8-h photoperiod for 9 days. Seedlings were then transferred to soil and grown in the same temperature and light conditions to analyze phenotype.

To measure BL inhibition of root growth, seeds were sterilized with 100% ethanol and germinated on MS plates containing the indicated BL concentration. After 2 days at 4°C for stratification, the seeds were grown vertically under long day conditions (16 h light/8 h dark) at 25°C. After 5 days, root length was measured and expressed as a percentage of the control length.

### SITE-DIRECTED MUTAGENESIS OF Flag-BAK1 CYTOPLASMIC DOMAIN AND RECOMBINANT PROTEIN STUDIES

After sequencing to confirm mutated regions, BAK1-CD and its mutations were expressed in BL21 (DE3) pLysS cells (Novagen, Gibbstown, NJ, USA). Cultures were induced with 0.3 mM IPTGat 25°C for 16 h and the soluble recombinant protein produced was purified using anti-Flag M2 affinity gel (Sigma-Aldrich, St. Louis, MO, USA). After elution from the beads, the protein solution was dialyzed against a 1000X volume of buffer containing 20 mM MOPS, pH 7.5, and 1 mM DTT. The ability of Flag-BAK1 and (wild type and C-terminal truncation mutant) to transphosphorylate Flag-BRI1 and increase its kinase activity was monitored using the BR13 peptide (sequence: GRJKKIASVEJJKK, where J is norleucine; produced by Bethyl Laboratories, Montgomery, TX, USA) as substrate as previously described using the filter binding assay (Wang et al., 2008).

### PREPARATION OF MICROSOMAL MEMBRANES AND IMMUNOPURIFICATION OF BAK1-Flag

Microsomal membranes were isolated from harvested tissues (Oh et al., 2009b), solubilized with Triton X-100, and incubated with anti-Flag M2 affinity gel at 4°C overnight with shaking. After incubation, anti-Flag M2 affinity beads were washed once with IPDB solution [20 mM MOPS (pH 7.5), 1 mM DTT, 1 mM EDTA, 4 mM NaF, 0.1 μM MCLR, 0.2 mM AEBSF, 0.2 mM BZ-HCl, 0.2 mM CA, 0.4 μM E64, 0.1% TritonX-100, and 10 mM MgCl_2_]; twice with PBS150 [5 mM NaP, 150 mM NaCl); once with PBS50 (5 mM NaP, 50 mM NaCl); and finally two washes with IPDB solution. After the final wash step, an aliquot of 1.5X SDS buffer was added and the mixture was heated at 95°C for 5 min to elute BAK1-Flag and BAK1-ΔCT-Flag proteins. Recombinant Flag-BAK1 was immunopurified using anti-Flag M2 affinity gel (Sigma, St. Louis, MO, USA) as previously described (Wang et al., 2005a, 2008).

RETRACTED

### IMMUNOBLOT ANALYSIS

Immunoprecipitated full-length BAK1-Flag or recombinant Flag-BAK1 proteins were subjected to SDS-PAGE followed by transfer to PVDF membranes and immunoblot analysis using anti-Flag antibodies (1:5,000 dilution), anti-phosphothreonine antibodies (1:500 dilution), and anti-phosphotyrosine antibodies (1:500 dilution). Immunoblots were scanned using an Odyssey Infrared Imaging System (LI-COR Bioscience, Lincoln, NE, USA) for visualization. Blots stained with ProQ Diamond phosphoprotein stain (Invitrogen, Carlsbad, CA, USA) were scanned using a Typhoon Molecular Dynamics phosphor/fluorescence imager.

### PEPTIDE INTERACTIONS STUDIES

The real-time binding of Flag-BRI1 (analyte) to immobilized BAK1 C-terminal domain peptides was monitored using an Octet QK (Pall ForteBio Corp, Menlo Park, CA, USA). The binding buffer contained 50 mM MOPS (pH 7.5), 0.01% (v/v) Triton X-100, 20 mM NaCl and 5 mM MgCl_2_ unless specified otherwise. Synthetic peptides corresponding to the C-terminal domain of BAK1 (residues 576–615) were produced with an N-terminal biotin group and either no additional modifications (CT), with phosphorylation of the Tyr-610 residue (CTpY610) or phosphorylation of the Ser-612 residue (CTpS612). All peptides were synthesized by GenScript Corp (Piscataway, NJ, USA). Biotinylated peptides were captured to SA Streptavidin Biosensors followed by binding of the analyte Flag-BRI1 from a 100 μg/mL solution or as otherwise noted. One-shot *K*_D_ was calculated based on the 1:1 model and the average *K*_D_ was extracted from binding results for four different concentrations of the analyte.

## RESULTS AND DISCUSSION

### THE JUXTAMEMBRANE AND C-TERMINAL DOMAINS REGULATE BAK1 KINASE TRANSPHOSPHORYLATION ACTIVITY AND SPECIFICITY

As an initial approach to study the role of flanking domains, we used the Flag-BAK1 cytoplasmic domain construct to produce a set of deletion mutants lacking the juxtamembrane (J) domain, the C-terminal domain, or both. All constructs had the kinase (K) domain with a Flag-epitope tag at the N-terminus (**Figure 1A**). Interestingly, only the constructs with the juxtamembrane domain (BAK1-JKC and BAK1-JK) had robust autophosphorylation on threonine and tyrosine residues (**Figure 1B**). By monitoring the phosphorylation of *E. coli* proteins during production of the recombinant protein kinases (Chou et al., 2012; Wu et al., 2012), we could also assess the effect of flanking domain removal on transphosphorylation activity. As shown in **Figure 1C**, recombinant BAK1 lacking the juxtamembrane domain was unable to transphosphorylate bacterial proteins on threonine or tyrosine residues, whereas constructs with the juxtamembrane were active. However, strongest transactivation was observed when the C-terminal domain was removed (BAK1-JK compared to BAK1-JKC; **Figure 1C**). Collectively, these results suggest that the juxtamembrane domain is an activator of the kinase domain, both in terms of auto- and trans-phosphorylation activity, and that the C-terminal domain is a strong inhibitor in particular of transphosphorylation activity. Alternatively, the C-terminal domain may affect specificity of the BAK1 kinase domain such that additional bacterial proteins and phosphorylation motifs are recognized when the C-terminal domain is truncated, which could also result in increased transphosphorylation activity. It will be important in future studies to distinguish between increased activity *per se* and altered specificity.

RETRACTED

**FIGURE 1:** **The juxtamembrane domain is a positive regulator while the C-terminal domain is a negative regulator of recombinant BAK1 transphosphorylation activity. (A)** Schematic representation of the Flag-BAK1-cytoplasmic domain truncations used in these experiments. J, K, and C, refer to the juxtamembrane, kinase, and C-terminal domains, respectively. Residue numbers at the domain interfaces are shown. **(B)** Autophosphorylation activity of the recombinant proteins measured with Pro-Q Diamond stain and immunoblotting with antiphosphotyrosine (pY) or antiphosphothreonine (pT) antibodies. Recombinant proteins were detected by immunoblotting with anti-Flag or peptide antibodies directed against the C-terminus of BAK1 (anti-BAK1; antigen sequence: DSTSQIENEYPSGPR_COOH_). Note the lack of cross reactivity of the anti-BAK1 antibodies with truncation mutants lacking the C-terminal domain. **(C)** Transphosphorylation of *E. coli* proteins that occurred during production of the BAK1 proteins shown in **(A)**. Phosphorylation of proteins was assessed as described in **(B)***, *except that proteins were visualized by staining with Coomassie Brilliant Blue (CBB).

Another interesting point is that the BAK1-JK truncation had strong autophosphorylation on tyrosine residues (**Figure 1B**). This was unexpected, because with the full-length BAK1 cytoplasmic domain protein, Tyr-610 in the C-terminal domain is a major site of autophosphorylation such that tyrosine autophosphorylation of the Y610F directed mutant is substantially reduced relative to the wild type protein (Oh et al., 2010). We predicted, therefore, that the BAK1-JK truncation mutant would have much reduced tyrosine autophosphorylation; however, that was not observed suggesting that additional tyrosine residues located in the kinase domain may be autophosphorylated in the absence of the C-terminal domain. To explore this possibility, we generated site-directed mutants by individually replacing each of the seven tyrosine residues in the kinase domain with phenylalanine. As expected from studies with the full-length cytoplasmic domain protein (Oh et al., 2010), Tyr-463 was also essential for kinase activity of the BAK1-JK truncation mutant as the Y463F directed mutant had strongly reduced autophosphorylation indicative of a kinase-inactive protein (**Figure 2**). The surprising result was that the Y304F and Y363F directed mutants had substantially reduced tyrosine autophosphorylation because in the full-length cytoplasmic domain proteins these substitutions have relatively little effect on the overall level of tyrosine autophosphorylation (Oh et al., 2010). Thus, Tyr-304 and Tyr-363 emerge as potential new sites of tyrosine autophosphorylation when the inhibitory C-terminal domain is removed. Threonine autophosphorylation was also increased when the C-terminal domain was truncated (**Figure 2**), but whether that was the result of autophosphorylation of new sites or increased stoichiometry of known sites is not clear and was not explored in the present study.

RETRACTED

**FIGURE 2:** **Effect of site-directed mutagenesis of kinase-domain tyrosine residues in Flag-BAK1-JK on autophosphorylation of the recombinant proteins. (A)** Autophosphorylation status as measured with Pro-Q Diamond stain and immunoblotting with antiphosphotyrosine (pY) or antiphosphothreonine (pT) antibodies. Recombinant proteins were detected by immunoblotting with anti-Flag antibodies. **(B)** Densitometry analysis of immunoblots shown in **(A)**. Phosphoamino acid signals are normalized with the amount of recombinant protein, determined by cross reaction with anti-Flag antibodies.

As an initial approach to determine which regions of the C-terminal domain are crucial to the transphosphorylation activity of BAK1, we constructed a nested series of truncations that sequentially removed five amino acid segments from the C-terminus of this flanking region (**Figure 3**). The full-length Flag-BAK1 cytoplasmic domain ends at residue 615 and only weakly transphosphorylates bacterial proteins on tyrosine and threonine relative to the BAK1-JK truncation mutant, which ends at residue 577. Removal of the last five residues of the C-terminal domain (to generate the CT610 mutant), substantially increased transphosphorylation activity on tyrosine and threonine residues, whereas the full effect required removal of the last twenty residues. Longer deletions beyond the CT595 truncation did not result in any further increase in transphosphorylation activity. These results suggest that the last half of the C-terminal domain is responsible for inhibition of transphosphorylation activity, possibly by interacting with the kinase domain and restricting protein substrate access to the active site.

RETRACTED

**FIGURE 3:** **Identification of residues in the C-terminal domain responsible for inhibition of BAK1 transphosphorylation activity. (A)** Serial deletions of the C-terminal domain were constructed to produce truncation mutants ending with the indicated residue. **(B)** Analysis of transphosphorylationof the C-terminal truncation mutants by immunoblotting with antibodies as described in the **Figure 1** legend.

### PLANT GROWTH IS REDUCED BY EXPRESSION OF A TRUNCATED BAK1 LACKING THE C-TERMINAL DOMAIN

In general, expressing a hyper-activated form of a receptor kinase would be expected to increase signaling *in vivo*. With BR signaling, increased plant growth would be expected and indeed was observed with plants expressing BRI1 lacking the inhibitory C-terminal domain (Wang et al., 2005b). Consequently, we anticipated that plants expressing the BAK1-ΔCT-Flag truncation mutant (**Figure 4A**) would have increased signaling and enhanced growth; however, that result was not obtained. As shown in **Figure 4B**, the BAK1-ΔCT-Flag plants had smaller roots when grown as seedlings on agar plates and the rosettes remained substantially smaller than plants expressing full-length BAK1-Flag during both vegetative and reproductive development (**Figure 4C**). Expression levels of the BAK1-ΔCT protein varied among transgenic lines tested but were not responsible for the reduced growth phenotype (**Figure 4D**). Moreover, both BAK1-Flag and BAK1-ΔCT-Flag were associated with BRI1 *in vivo*, as the two proteins were co-immunoprecipitated from all transgenic lines. Thus, the reduced growth was not the result of impaired binding of BAK1-ΔCT to BRI1 *in vivo*. Although growth of the BAK1-ΔCT-Flag plants was markedly reduced, rosette morphology was not indicative of impaired BR signaling as petioles and leaves were relatively elongated unlike strong BR signaling mutants (Clouse and Sasse, 1998).

**FIGURE 4:** **The C-terminal domain of BAK1 is required for normal vegetative and reproductive growth of *Arabidopsis*. (A)** Schematic representation of the constructs used to generate transgenic plants in the null *bak1bkk1* mutant background. **(B)** Root growth for seedlings on agar plates growing in the light. **(C)** Reduced growth of transgenic plants expressing BAK1-ΔCT-Flag compared to BAK1-Flag during vegetative and reproductive growth. **(D)** BRI1 protein co-immunoprecipitates with BAK1-Flag or BAK1-ΔCT-Flag.

RETRACTED

In an attempt to determine the basis for the strong phenotype of the transgenic plants expressing BAK1-ΔCT-Flag, we examined the ability of recombinant GST-BAK1-JK truncation mutant to transactivate BRI1 *in vitro*, which mimics their interaction *in vivo* and is thought to be essential for enhanced BR signaling *in vivo* (Wang et al., 2008). This functional interaction can be examined *in vitro* by monitoring the ability of BAK1 to increase the peptide kinase activity of BRI1using the SP11 synthetic peptide as substrate (Oh et al., 2000; Wang et al., 2008). As shown in **Figure 5** and as expected, Flag-BRI1 readily phosphorylated the SP11 synthetic peptide whereas GST-BAK1 or the GST-BAK1-JK truncation mutant did not. In addition, neither of the kinase inactive mutants (Flag-mBRI1 and GST-mBAK1) displayed peptide kinase activity. However, GST-BAK1 substantially increased the ability of Flag-BRI1to transphosphorylate the synthetic peptide substrate whereas the GST-BAK1-JK truncation mutant did not (**Figure 5**). As expected, the kinase-inactive GST-mBAK1 did not stimulate BRI1 peptide kinase activity because BAK1 kinase activity is required for the transphosphorylation/activation of BRI1 (Wang et al., 2008). It is important to note that the inability of GST-BAK1-JK to activate BRI1 is not the result of impaired kinase activity, as the C-terminal domain truncation mutant is active. The important conclusion is thatBAK1 C-terminal domain is required to fully activate BRI1, which is recognized to be an important factor that regulates signaling leading to plant growth (Vert et al., 2005; Oh et al., 2009a; Clouse, 2011).

**FIGURE 5:** **Activation of Flag-BRI1peptide kinase activity by GST-BAK1 but not GST-BAK1-JK or the kinase-inactive GST-mBAK1 directed mutant monitored using the SP11 synthetic peptide substrate.** The increase in BRI1 activity requires an active BAK1 kinase with C-terminal domain, which alone does not readily phosphorylate the SP11 peptide. Values are means ± SEM; *n* = 3.

The above results suggest that reduced growth in the BAK1-ΔCT-Flag plants may be the result of attenuated BR signaling. To test this notion, we examined the inhibition of root elongation by high concentrations of BL (Clouse et al., 1996; Li et al., 2001). As shown in **Figure 6**, concentrations of brassinolide above 1 nM inhibited root elongation in the wild type BAK1-Flag plants to a much greater extent than the *bri1-5* plants, which is consistent with the reduced BR signaling in the *bri1-5* plants. Root elongation in the BAK1-ΔCT-Flag plants was inhibited by BL but to a lesser extent than in plants expressing wild type BAK1-Flag. These results suggest that BR signaling was somewhat reduced by truncation of the C-terminal domain of BAK1, but perhaps cannot completely explain the reduction in plant growth. It is possible that growth is restricted as a combination of reduced BR signaling and other factors that remain to be identified.

RETRACTED

**FIGURE 6:** **Inhibition of root elongation by high concentrations of BL.** Root elongation in *bri1-5* plants is relatively insensitive to BL as a result of impaired BR signaling. Transgenic plants expressing BAK1-ΔCT-Flag are slightly less sensitive to BL compared to BAK1-Flag plants suggesting that truncation of BAK1 results in some reduction in BR signaling.

One potential factor for the reduced growth phenotype of BAK1-ΔCT-Flag plants could be activation of defense mechanisms, which often results in growth inhibition (Zhu et al., 2013). This might occur, for example, as the result of activation of FLS2 when the hyperactivated BAK1-ΔCT-Flag protein is expressed. Alternatively, removal of the C-terminal domain of BAK1 may alter specificity of the kinase domain rather than activity *per se*. As mentioned above, the increased transphosphorylation activity observed in *E. coli* (**Figure 1C**) may reflect altered specificity (rather than increased activity) that allows the recombinant Flag-BAK1-JK protein to phosphorylate a broader array of bacterial proteins. If this broadened specificity occurred in planta, it may result in inappropriate signaling causing growth inhibition. We will test these possibilities in future experiments by analyzing gene expression in BAK1-ΔCT-Flag plants to ascertain whether defense genes are activated in the absence of (apparent) external triggers. We will also determine whether levels of FLS2 protein are reduced, as FLS2 degradation follows its activation (Robatzek et al., 2006). A third possibility that may explain altered signaling by BAK1-ΔCT-Flag is that the protein has altered subcellular localization. At present we have no information about this aspect, but in future studies will attempt to examine this using a GFP-tagged construct.

### BINDING OF THE BAK1 C-TERMINAL DOMAIN TO BRI1

The observation that removal of the C-terminal domain of BAK1 enhances transphosphorylation activity *in situ* but prevents the proper activation of BRI1 *in vitro* suggests that the C-terminal domain may play a specific role in the correct positioning of BAK1 with BRI1 (at least *in vitro*). One possibility would be that when the two receptor kinases are juxtaposed, the C-terminal domain of BAK1 binds to BRI1, thereby helping to properly position the two kinase domains while also relieving the inhibitory effect of the C-terminal domain on BAK1 transphosphorylation activity. To test this notion, we asked whether recombinant Flag-BRI1 would bind to the immobilized C-terminal polypeptide of BAK1. As shown in **Figure 7A**, with a synthetic peptide based on the entire C-terminal domain of BAK1 (residues 576 to 615; designated CT in **Figure 7**) as the immobilized ligand, recombinant Flag-BRI1 protein (analyte) interacted but only weakly. However, robust binding of Flag-BRI1 was observed with the C-terminal domain peptide phosphorylated at the Tyr-610 site (designated CTpY610 in **Figure 7**). The increased binding could not be attributed simply to adding negative charge to the polypeptide because the CT peptide phosphorylated at the Ser-612 site (designated CTpS612) only supported slightly more binding than the unphosphorylated CT peptide (**Figure 7**). Binding of Flag-BRI1 to the CTpY610 peptide increased as pH of the reaction mixture was reduced from pH 8–7, but binding to the immobilized CT peptide was low and constant over the same pH range (**Figure 7B**). Interestingly, early studies (Oh et al., 2000) with recombinant Flag-BRI1 found that both autophosphorylation and transphosphorylation (peptide kinase) activity had a pH optimum near 7.0, which is similar to the results of the present study. It is conceivable that pH is affecting BRI1 overall conformation or the charge of specific groups on the surface of the molecule, but effects on the charge of the CT peptide could also be involved. It is also worth noting that robust binding of Flag-BRI1 to the CTpY610 peptide also required Mg^2^^+^; in the absence of the divalent cation binding to the CT or CTpY610 was completely prevented (**Figure 7B**). It is recognized that many protein kinases, such as protein kinase A (Adams and Taylor, 1993; Bastidas et al., 2013) bind divalent cations with dramatic effects on kinase activity and conformational changes could certainly be involved. In support of that notion, earlier work demonstrated that binding of Flag-BRI1 to immobilized GST-BAK1 was completely dependent on Mg^2^^+^ (Oh et al., 2010). The Mg^2^^+^-dependence of binding in both systems suggests that the interactions are specific and that “active” conformations of the kinases are required. Future studies will determine whether divalent cation induced conformational changes occur and are responsible for the enhanced binding. Greatest binding of Flag-BRI1 to the immobilized CTpY610 peptide occurred at pH 7.0 with Mg^2^^+^ in the reaction mixture, and under these conditions a *K*_D_ for binding of ~34 ± 3 nM was estimated (**Figure 7C**), which is similar to the affinity of the interaction between GST-BAK1 and Flag-BRI1 *in vitro* (Oh et al., 2010).

RETRACTED

**FIGURE 7:** **Label-free binding of recombinant BRI1 protein to an immobilized peptide based on the BAK1 C-terminal domain sequence (residues 576–615).** Binding was monitored in the Octet, which uses fiber optic sensors to detect protein-protein or protein-peptide interactions using biolayer interferometry. **(A)** Phosphorylation of the Tyr-610 residue (CTpY610) supports robust binding of Flag-BRI1 compared to phosphorylation of the Ser-612 site (CTpS612) or the unphosphorylated peptide (CT). All reactions were run at pH 7.0. **(B)** Binding of Flag-BRI1 to the CTpY610 peptide is sensitive to pH and is strictly dependent on Mg^2^^+^, whereas binding to the CT peptide is low, shows no pH dependence, but is also strictly dependent on Mg^2^^+^. **(C)** Binding of various concentrations of Flag-BRI1 to the immobilized CTpY610 peptide to estimate the binding affinity.

## CONCLUSION

Our results support a model that involves inhibition of BAK1 kinase activity by its C-terminal domain, which we postulate can be relieved by its binding to the cytoplasmic domain of BRI1 after formation of the BRI1:BAK1 complex. Interestingly, the flanking domains of BRI1 (Oh et al., 2009b, 2012) and BAK1 (this study) have similar effects on kinase activity, with the juxtamembrane domains activating while the C-terminal domains inhibit kinase activity. In the case of BRI1, inhibition by the C-terminal domain is relieved by autophosphorylation of residues within the domain and expression of a BRI1-ΔCT truncation mutant in transgenic plants results in hyper-activation of BR signaling and increased plant growth (Wang et al., 2005b). In contrast, inhibition by the C-terminal domain of BAK1 is not relieved solely by autophosphorylation and expression of BAK1-ΔCT-Flag in transgenic plants does not hyperactivate signaling and actually results in reduced plant growth. The growth inhibition cannot be completely attributed to reduced BR signaling (**Figure 5B**), which is also supported by the observation that plants do not have the morphology of BR signaling mutants (**Figure 4C**). We speculate that other factors may be involved in reducing plant growth, such as enhanced stress signaling in plants expressing BAK1-ΔCT-Flag, perhaps as a result of FLS2 activation, or inappropriate signaling that occurs as a result of altered specificity of the BAK1-ΔCT-Flag protein. These are important questions but are beyond the scope of the present study. Much also remains to be done with the possible role of the C-terminal domain of BAK1 in its interaction with BRI1 resulting in BR signaling. In particular, it will be interesting to determine whether C-terminal domain binding between proteins applies to other receptor:co-receptor kinase pairs as well. Our present results are generally consistent with the previous report that C-terminal epitope tags can affect BAK1 function in different signaling pathways (Ntoukakis et al., 2011). Our results extend this concept to establish a role for the C-terminal domain itself at least with BAK1 as co-receptor with BRI1 in BR signaling. Because BAK1 also serves as co-receptor with the leucine-rich repeat receptor kinases flagellin-sensitive 2 (FLS2) and elongation factor TU receptor (EFR; Chinchilla et al., 2007), it will be interesting to determine whether the C-terminal domain of BAK1 is essential for these signaling pathways and we will explore this in future studies.

RETRACTED

## Conflict of Interest Statement

The authors declare that the research was conducted in the absence of any commercial or financial relationships that could be construed as a potential conflict of interest.
